The article "Vesicourachal Diverticulum: A Rare Cause of Recurrent Urinary Tract Infections" was retracted in 2024. Reasons: false authorship; unreliable results or conclusions; no approval from an author; concerns about the authorship.

# Vesicourachal Diverticulum: A Rare Cause of Recurrent Urinary Tract Infections

**DOI:** 10.7759/cureus.20118

**Published:** 2021-12-02

**Authors:** Mohammed A Alqarni, Rahmah H Kutubkhana, Sara M Alhosami, Faris A Almutairi, Amer M Almutairi, Edris M Alqannad, Mohammed H Almansour, Abrar A Alanazi, Abdulaziz M Althobaiti, Ziyad F Althobaiti, Mohammed A Alshehri, Sulaiman Z Malki, Hussain M Alhasani, Mohammed A Alburi, Faisal Al-Hawaj

**Affiliations:** 1 College of Medicine, King Saud University, Riyadh, SAU; 2 College of Medicine, Batterjee Medical College, Jeddah, SAU; 3 College of Medicine, Ibn Sina National College for Medical Studies, Jeddah, SAU; 4 College of Medicine, King Saud Bin Abdulaziz University for Health Sciences, Riyadh, SAU; 5 General Practice, King Faisal Hospital, Mecca, SAU; 6 College of Medicine, Najran University, Najran, SAU; 7 College of Medicine, Tabuk University, Tabuk, SAU; 8 College of Medicine, Taif University, Taif, SAU; 9 College of Medicine, Taibah University, Medina, SAU; 10 College of Medicine, Umm Al-Qura University, Mecca, SAU; 11 College of Medicine, Vision Colleges, Riyadh, SAU; 12 College of Medicine, Imam Abdulrahman Bin Faisal University, Dammam, SAU

**Keywords:** case report, computed tomography, vesicourachal diverticulum, urachal anomalies, recurrence, urinary tract infection

## Abstract

Urinary tract infection is a common medical condition encountered in outpatient clinics and emergency departments. Recurrence of urinary tract infections is common. The recurrence can arise from behavioral, mechanical, and physiological factors. Urachal anomalies are very rare congenital clinical entities. We present the case of a 41-year-old woman who presented to the emergency department with dysuria, frequency, urgency, and incontinence. There was no history of fever or flank pain. Physical examination revealed no abnormalities. Initial laboratory markers were within the normal range. However, urinalysis findings showed numerous white blood cells and positive leukocyte esterase and nitrite. While these findings are suggestive of acute simple cystitis, the patient had a concerning history of recurrent urinary tract infections. The urology team advised performing an abdominal computed tomography scan to rule out any structural abnormalities. The patient underwent a computed tomography scan, which demonstrated the presence of a fluid-filled structure arising from the dome of the bladder and extending superiorly toward the umbilicus, representing a vesicourachal diverticulum. The patient underwent surgical resection after antibiotic therapy. The vesicourachal diverticulum is a very rare type of urinary tract anomalies. The case highlights the importance of considering congenital urachal anomalies in patients with recurrent urinary tract infections. A computed tomography scan can make the diagnosis of such anomalies with high accuracy.

The article "Vesicourachal Diverticulum: A Rare Cause of Recurrent Urinary Tract Infections" was retracted in 2024. Reasons: false authorship; unreliable results or conclusions; no approval from an author; concerns about the authorship.

## Introduction

Urinary tract infections are the most common infections encountered in the outpatient department [1]. The lifetime prevalence of urinary tract infections in women exceeds 50%. Most urinary tract infections are acute simple cystitis rather than acute pyelonephritis [2]. Recurrence is common with urinary tract infections. The recurrence typically results from reinfection rather than a relapse due to incomplete eradication of the prior infection [3]. The majority of women with recurrent urinary tract infections do not undergo further imaging or urologic evaluation. The proposed risk factors for recurrent urinary tract infections include behavioral, mechanical, and physiological risk factors [2]. The behavioral risk factors include factors related to the sexual activity such as the use of spermicides. Physiological factors include the estrogen deficiency status in postmenopausal women [4]. However, factors that influence bladder emptying were found to be strongly associated with the recurrence of infections. Here, we present the case of a middle-aged woman with a history of recurrent urinary tract infections, which was found to result from vesicourachal diverticulum, a form of congenital urachal anomalies.

## Case presentation

We present the case of a 41-year-old woman who presented to the emergency department with urinary frequency and urgency for the last 3 days. She reported that she had an abrupt compelling desire to pass urine that she cannot defer. This was often associated with loss of urinary control. The urination was associated with a burning sensation. The patient reported that needs to pass urine every 3 hours and she woke up more than once at night to urinate. There was no change in the urine color. The patient did not report any history of flank pain or fever.

The patient had a significant medical history of recurrent urinary tract infections. Approximately, she developed cystitis every 5 months for the last 15 years. She was known to have asthma and beta-thalassemia minor. Her surgical history was remarkable for transsphenoidal hypophysectomy performed 10 years ago for pituitary adenoma. The patient was a heavy smoker (30 pack-years) but never consumed alcohol. She worked as a taxi driver. Her family history was non-contributory.

Upon examination, the patient did not appear in distress. Her vital signs included a heart rate of 90 bpm, respiratory rate of 14 bpm, the temperature of 37.0℃, and blood pressure of 110/78 mmHg. Her oxygen saturation was normal on room air. Abdominal examination showed no tenderness or rigidity. The bowel sound was audible with normal intensity and frequency. Examination of other systems was non-contributory.

The article "Vesicourachal Diverticulum: A Rare Cause of Recurrent Urinary Tract Infections" was retracted in 2024. Reasons: false authorship; unreliable results or conclusions; no approval from an author; concerns about the authorship.

Initial laboratory markers revealed a hemoglobin level of 14.2 g/dL, leukocytes count of 5200/μL, and platelets count of 380,000/μL. The inflammatory parameters, including erythrocyte sedimentation rate and C-reactive protein, were within the normal limits (Table 1). Urinalysis findings showed numerous leukocytes with positive leukocyte esterase and nitrite. Despite the recurrent history of urinary tract infection, the patient had not undergone any imaging studies previously. The urology team advised performing an abdominal computed tomography scan to rule out any structural abnormalities.

**Table 1:** Summary of the results of laboratory findings

Laboratory Investigation	Unit	Result	Reference Range
Hemoglobin	g/dL	14.2	13.0–18.0
Leukocytes	1000/mL	5200	4.0–11.0
Platelet	1000/mL	380	140–450
Erythrocyte Sedimentation Rate	mm/h	14	0–20
C-Reactive Protein	mg/dL	5.8	0.3–10.0
Total Bilirubin	mg/dL	0.8	0.2–1.2
Albumin	g/dL	4.5	3.4–5.0
Alkaline Phosphatase	U/L	52	46–116
Gamma-glutamyltransferase	U/L	18	15–85
Alanine Transferase	U/L	20	14–63
Aspartate Transferase	U/L	22	15–37
Blood Urea Nitrogen	mg/dL	9	7–18
Creatinine	mg/dL	0.9	0.7–1.3
Sodium	mEq/L	138	136–145
Potassium	mEq/L	3.9	3.5–5.1
Chloride	mEq/L	104	98–107

The patient underwent a contrast-enhanced computed tomography scan, which demonstrated the presence of a fluid-filled structure arising from the dome of the bladder and extending superiorly toward the umbilicus. Such findings conferred the diagnosis of vesicourachal diverticulum, a type of congenital urachal anomalies (Figures 1, 2).

**Figure 1:** Axial CT image demonstrates an outpouching fluid-filled structure (arrow) arising from the dome of the bladder. CT: computed tomography

**Figure 2:** Sagittal CT image demonstrates a fluid-filled structure (arrow) extending superiorly from the bladder toward the umbilicus. CT: computed tomography

The patient was given cefuroxime for the management of her current cystitis. After completion of the antibiotic course and having a negative bacterial culture, surgical management for the anomaly was planned. The patient underwent laparotomy for the resection of the urachal diverticulum. The operation was successful with no complications. The patient had an uneventful recovery. She was discharged on the fourth postoperative day. After 6 months of follow-up visits, the patient remained asymptomatic and had no further infections.

## Discussion

We report the case of recurrent urinary tract infections resulting from a congenital anatomic anomaly in the urinary tract [5]. The urachus is an embryonal remnant of the allantois and it is a midline tubular structure connecting the bladder to the umbilicus. Normally, the urachus undergoes involution before birth and forms the median umbilical ligament. Failure of the involution results in a spectrum of anomalies that include patent urachus, urachal sinus, vesicourachal diverticulum, and urachal cyst [6]. In the present case, the patient was found to have vesicourachal diverticulum, which is the rarest type of congenital urachal anomalies [7].

The article "Vesicourachal Diverticulum: A Rare Cause of Recurrent Urinary Tract Infections" was retracted in 2024. Reasons: false authorship; unreliable results or conclusions; no approval from an author; concerns about the authorship.

Regarding the clinical manifestations of urachal anomalies, the majority of cases are asymptomatic and found incidentally on cross-sectional imaging studies performed for other indications. As in the present case, urachal anomalies may result in infections [8]. Since urinary tract infections are common among women, these patients tend not to have any further workup or imaging studies even if they have frequent recurrent infections [6]. Malignancy is the other important complication of urachal anomalies. The malignant tumors arising from the urachal anomalies do not tend to be transitional cell carcinoma.

It is common for urachal anomalies to be confused with a wide range of conditions. Such conditions include acute appendicitis, endometriosis, ovarian torsion, and incarcerated hernia [7]. Imaging studies can readily make the diagnosis of urachal anomalies [6]. In the present case, the treating physician suspected some anatomic anomalies in the patient causing the history of recurrent urinary tract infections and requested a computed tomography scan to identify such anomaly.

Surgical resection of the urachal anomalies is the treatment of choice. However, the surgery should be conducted after the infection is eradicated with broad-spectrum antibiotics [6]. This is essential to reduce the risk of postoperative complications like surgical-site infections. In the present case, the surgery was performed after obtaining a negative culture following antibiotic therapy. The excision of the urachal remnant can be done as a one-stage or two-stage procedure. In the two-stage procedure, the first operation involves incision and drainage of the remnant followed by a second operation to excise the remnant [9].

## Conclusions

The vesicourachal diverticulum is a very rare type of urinary tract anomalies. The case highlights the importance of considering congenital urachal anomalies in patients with recurrent urinary tract infections. Physicians should consider the possibility of anatomic anomalies in patients with recurrent urinary tract infections. A computed tomography scan can make the diagnosis of such anomalies with high accuracy. Early diagnosis and management of such anomalies in symptomatic patients can reduce the morbidity of patients because of frequent hospital visits due to recurrent infections.

The article "Vesicourachal Diverticulum: A Rare Cause of Recurrent Urinary Tract Infections" was retracted in 2024. Reasons: false authorship; unreliable results or conclusions; no approval from an author; concerns about the authorship.

## References

[1] McLellan LK, Hunstad DA (2016). Urinary tract infection: pathogenesis and outlook. Trends Mol Med.

[2] Nicolle LE (2008). Uncomplicated urinary tract infection in adults including uncomplicated pyelonephritis. Urol Clin North Am.

[3] Wagenlehner FM, Weidner W, Naber KG (2009). An update on uncomplicated urinary tract infections in women. Curr Opin Urol.

[4] Butler CC, Francis N, Thomas-Jones E (2017). Variations in presentation, management, and patient outcomes of urinary tract infection: a prospective four-country primary care observational cohort study. Br J Gen Pract.

[5] Walker C (2010). A case report of urachal abscess: a rare differential in adult abdominal pain. Hawaii Med J.

[6] Jayakumar S, Darlington D (2020). Acute presentation of urachal cyst: a case report. Cureus.

[7] Parada Villavicencio C, Adam SZ, Nikolaidis P, Yaghmai V, Miller FH (2016). Imaging of the urachus: anomalies, complications, and mimics. Radiographics.

[8] Yu JS, Kim KW, Lee HJ, Lee YJ, Yoon CS, Kim MJ (2001). Urachal remnant diseases: spectrum of CT and US findings. Radiographics.

[9] Elkbuli A, Kinslow K, Ehrhardt JD Jr, Hai S, McKenney M, Boneva D (2019). Surgical management for an infected urachal cyst in an adult: case report and literature review. Int J Surg Case Rep.

